RETRACTED

# Combination of mTOR and EGFR Kinase Inhibitors Blocks mTORC1 and mTORC2 Kinase Activity and Suppresses the Progression of Colorectal Carcinoma

**DOI:** 10.1371/journal.pone.0073175

**Published:** 2013-08-22

**Authors:** Quan Wang, Feng Wei, Chunsheng Li, Guoyue Lv, Guangyi Wang, Tongjun Liu, Anita C. Bellail, Chunhai Hao

**Affiliations:** 1 Department of Gastrointestinal Surgery, First Hospital of Jilin University, Changchun, Jilin, China; 2 Department of Hepatopancreatobiliary Surgery, First Hospital of Jilin University, Changchun, Jilin, China; 3 Department of Colorectal Surgery, Third Hospital of Jilin University, Changchun, Jilin, China; 4 The Department of Pathology & Laboratory Medicine, Emory University, Atlanta, Georgia, United States of America; Boston University Goldman School of Dental Medicine, United States of America

## Abstract

Mammalian target of rapamycin complex 1 and 2 (mTORC1/2) are overactive in colorectal carcinomas; however, the first generation of mTOR inhibitors such as rapamycin have failed to show clinical benefits in treating colorectal carcinoma in part due to their effects only on mTORC1. The second generation of mTOR inhibitors such as PP242 targets mTOR kinase; thus, they are capable of inhibiting both mTORC1 and mTORC2. To examine the therapeutic potential of the mTOR kinase inhibitors, we treated a panel of colorectal carcinoma cell lines with PP242. Western blotting showed that the PP242 inhibition of mTORC2-mediated AKT phosphorylation at Ser 473 (AKT^S473^) was transient only in the first few hours of the PP242 treatment. Receptor tyrosine kinase arrays further revealed that PP242 treatment increased the phosphorylated epidermal growth factor receptor (EGFR) at Tyr 1068 (EGFR^T1068^). The parallel increase of AKT^S473^ and EGFR^T1068^ in the cells following PP242 treatment raised the possibility that EGFR phosphorylation might contribute to the PP242 incomplete inhibition of mTORC2. To test this notion, we showed that the combination of PP242 with erlotinib, an EGFR small molecule inhibitor, blocked both mTORC1 and mTORC2 kinase activity. In addition, we showed that the combination treatment inhibited colony formation, blocked cell growth and induced apoptotic cell death. A systemic administration of PP242 and erlotinib resulted in the progression suppression of colorectal carcinoma xenografts in mice. This study suggests that the combination of mTOR kinase and EGFR inhibitors may provide an effective treatment of colorectal carcinoma.

## Introduction

Colorectal carcinoma is the third most common cancer in men and women but the second leading cause of cancer-related deaths in the United States [1]. Recent advances in research suggest that targeting of mTOR pathway may provide novel therapies for clinical treatment of the carcinoma [2]. The mTOR is a conservative serine/threonine (S/T) protein kinase of the phosphatidylinositol 3-kinase (PI3K) family [3]. The mTOR kinase exists in two functional complexes: mTOR complex 1 (mTORC1) and mTOR complex 2 (mTORC2) [4]. Both the complexes contain the mTOR kinase but they are distinguished by unique regulatory proteins: the regulatory-associated protein of mTOR (RAPTOR) defines mTORC1 [5] whereas the rapamycin-insensitive companion of mTOR (RICTOR) is specific to mTORC2 [6]. The mTORC1 controls the rate of protein synthesis through phosphorylation and activation of its substrates, p70S6 ribosomal kinase 1 (p70S6K) and eukaryotic translation initiation factor 4E (eIF4E) binding protein-1 (4E-BP1) and once phosphorylated, p70S6K phosphorylates ribosomal protein S6 and 4E-BP1 becomes dissociated from eIF4 and promote mRNA translation and protein synthesis [7]. On the other hand, mTORC2 regulates cell survival and cell cycle progression through phosphorylation of AKT, serum- and glucocorticoid-regulated kinase (SGK) and protein kinase C (PKC) [8–11].

mTOR is a central integrator for upstream inputs from growth factors, nutrients and stress [12]. Insulin-like growth factor-1 (IGF1), for instance, can activate mTORC1 through its receptor tyrosine kinase (RTK)-mediated phosphorylation and activation of PI3K and AKT and AKT in turn mediates phosphorylation of tuberous sclerosis 2 (TSC2) and proline-rich AKT substrate 40 kDa (PRAS40), thus releasing their inhibition of mTORC1 [13,14]. RTKs also activate mTORC1 through Ras-extracellular signal-regulated kinase (ERK) pathway [15] and subsequent ERK phosphorylation of the mTORC1 inhibitor TSC2 [16] and RAPTOR [17]. This growth factor-mTORC1 pathway is regulated through two negative feedback loops: mTORC1-p70S6K-mediated phosphorylation and degradation of insulin receptor substrate (IRS) [18,19] and mTORC1-mediated phosphorylation of growth factor receptor-bound protein 10 (GRB10) [20].

RETRACTED

The mTOR pathway is overactive in cancers [21]; thus, mTOR inhibitors have been developed as cancer therapeutic agents [22,23]. The first generation of mTOR inhibitors, rapamycin and its analogs (known as rapalogs) such as everolimus (RAD001), temsirolimus (CCI-779) and ridaforolimus (AP23573) have entered clinical trials but, unfortunately, shown limited clinic benefits against many types of cancers [24,25], even though temsirolimus has been approved for clinical treatment of renal cell carcinoma in United States [26]. Patients with advanced carcinoma, for instance, show a partial response to rapalog treatment in phase I trials [27,28]. The cancer resistance to the rapalog treatment is mainly due to the existence of negative feedback loops. Rapamycin interacts with FK506 binding protein 12 (FKBP-12) and form a complex that binds and removes RAPTOR from mTORC1 [29]; thus, rapamycin inhibits mTORC1 but has little effect on mTORC2. By inhibiting mTORC1, rapalog prevents inhibitory IRS phosphorylation and degradation and activates PI3K/AKT [30,31] and ERK pathway through the feedback loops [32–34]. In addition, rapalogs incompletely inhibit the 4E-BP1 phosphorylation [35] and do not induce apoptosis in cancer cells [36] because the IGF1 pathway inhibits apoptosis [37].

The second generation of mTOR inhibitors has been developed to target the adenosine triphosphate (ATP)-binding site of mTOR kinase [38]. These mTOR kinase inhibitors such as Torin1, PP242 and PP30 block p70S6K, 4E-BP1 and AKT phosphorylation and thus inhibit both mTORC1 and mTORC2 [39,40]. In addition, Torin1 activates autophagy in mammalian cells [39] whereas PP242 is cytotoxic [41] and induce apoptosis in leukemia and breast cancer cells through inhibition of mTORC2 activity [42,43]. Both mTORC1 and mTORC2 are active in colorectal carcinoma tissues [44–46]. Treatment of the carcinoma cell lines with PP242 inhibits the cell growth [47] and xenograft progression [48]. However, many of the cell lines are resistant to the PP242 treatment [48]. Another concern is inferred from the study of multiple myeloma cells, showing that, even though mTOR kinase inhibitors target mTORC1 and mTORC2, incomplete inhibition can lead to the loss of feedback inhibition of PI3K-AKT pathway [49].

To examine the therapeutic potential of the mTOR kinase inhibitor PP242, we show here that PP242 can only transiently block the mTORC2 kinase activity in the first few hours of the treatment. In parallel, the return of mTORC2 kinase activity is associated with the increase of phosphorylated EGFR. The combination treatment of PP242 and erlotinib, an EGFR inhibitor, completely block both mTORC1 and mTORC2 activity, inhibits cell growth and suppresses the progression of colorectal carcinoma xenografts.

## Materials and Methods

### Human colorectal carcinoma cell lines, tissues and normal colon tissues

Human colorectal carcinoma cell lines Caco_2_, Colo205, Colo320, DLD-1, HCT-8, HT29, HCT-116 and SW948 were purchased from American Type Collection (Rockville, MD) and grown in RPMI-1640 medium (Invitrogen, Carlsbad, CA) supplemented with 10% fetal bovine serum (FBS) and 1% penicillin-streptomycin in a humidified 5% CO_2_ and 37 ^o^C incubator. Matched colorectal carcinoma and normal colon tissue samples were collected in the First Hospital Tissue Bank. All patients provided written informed consent for tissue sample collection in the bank. This study was approved by the First Hospital Ethical Committee of Jilin University.

RETRACTED

### Reagents and antibodies

PP242 (Calbiochem, EMD Millipore), erlotinib, rapamycin and LY294002 (LC laboratories, Woburn, MA) were dissolved in dimethyl sulfoxide at the concentrations of 10 or 20 mM and stored in aliquots at -80^o^C. Epidermal growth factor (EGF) was purchased from Peprotech (RockyHillNJ). From Cell Signaling Technology (Beverly, MA) were the antibodies against human mTOR, phosphor-mTOR (Ser2448), AKT, phosphor-AKT (Ser473), S6, phophor-S6 (Ser235/236), 4E-BP1, phophor-4E-BP1 (Ser37/46), EGFR, phosphor-EGFR (Tyr1068). Also included in the study were the antibodies against DNF fragmentation factor (DFF45), poly (ADP-ribose) polymerase (PARP), caspase-3 (StressGen, Ann Arbor, MI), β-actin (Santa Cruz, CA), horseradish peroxidase (HRP)-conjugated goat anti-mouse and goat anti-rabbit antibodies (Jackson IR Laboratories, West Grove). Protease inhibitor mixture, Triton X-100 and other chemicals were from Sigma-Aldrich.

### Cell viability assay

Cells were seeded and grown in 96-well plates at 8ⅹ10^3^ cells per well in 100 ul of growth medium. Cells were treated or untreated with PP242 and erlotinib, alone or in combination. After incubation for the times indicated in the Results, cells were washed with a phosphate buffer and each of the wells was added with 100 ul buffer 0.2M containing sodium acetate (pH 5.5), 0.1% (v/v) Triton X-100 and 20 mM p-nitrophenyl phosphate. The plates were incubated at 37 ^o^C for 1.5 hours and the reaction was stopped by the addition of 10 ul 1M NaOH to each well and the color developed was measured at 405 nm by a microplate reader (BioRad).

### Colony formation assay

Cells in single-cell suspension were plated and grown in 6-wells plates at a density of 1000 cells per well for 24 hours. Cells were then treated or untreated with PP242 and erlotinib, alone or combination. The medium was replaced every 4 days with fresh medium containing PP242 and/or erlotinib. After 14 days, the medium was removed and cell colonies were stained with 0.5% crystal violet solution.

### Flow cytometric assay for sub-G1 apoptotic cells

Cells were treated with 1 uM PP242 and 2 uM erlotinib, alone or in combination, for 20 hours, harvested, fixed with 70% ethanol, and stained with propidium iodide. The data were acquired using a flow cytometry (FACSCanto II Becton Dickinson, Franklin Lakes, NY, USA) and were analyzed using FlowJo software (Tree Star Inc., Ashland, OR, USA). Sub-G1 apoptotic cells were presented in percentage of the cells.

RETRACTED

### Western blotting for protein expression and caspase cleavage

Western blotting was carried out based on the protocols reported earlier [50]. Cells were lysed in lysis a cell lysis buffer (20 nM Tris pH7.4, 150mM NaCL, 1% NP-40, 10% glycerol,1mM EGTA, 1mM EDTA, 5 mM sodium pyrophosphate, 50 mM sodium fluoride, 10 mM β-glycerophosphate, 1 mM sodium vanadate, 0.5 mM DTT, 1 mM PMSF, 2 mM imidazole, 1.15 mM sodium molybdate, 4mM sodium tartrate dihydrate, and 1ⅹ protease inhibitor cocktail). Cell lysates were cleared by centrifugation at 18,000 x g for 15 minutes at 4^o^C. The supernatant was collected and protein concentrations were determined by the Bradford protein assay following the manufacturer’s protocol (Bio-Rad Laboratories). Equal amounts of protein were separated through SDS-PAGE gels and transferred onto nitrocellulose membranes (Bio-Rad Laboratories). The membranes were incubated overnight at 4^o^C with primary antibody and then for 1 hour with HP-conjugated secondary antibody. The membranes were developed by chemiluminescence.

### Phosphorylated RTK Array

The pathScan RTK Signaling Antibody Array Kit was purchased from Cell Signaling Technology (Beverly, MA). This slide-based antibody array included twenty-eight RTKs. The slides were incubated with cell lysates and revealed by chemiluminescence according to the manufacturer’s instructions.

### Mouse subcutaneous xenografts and treatments

The animal studies were approved by the Institutional Animal Care and Use Committee of Emory University. The DLD-1 cells (7×10^6^) were injected subcutaneously into the flank regions of six-week old (about 20 g of body weight) female athymic (nu/nu) mice (Taconic, Hudson, NY). The mice were allowed to develop subcutaneous xenografts and tumor volumes were measured using caliper measurements. When tumors reached approximately 150-200 mm^3^, mice were assigned randomly to 3 experimental groups (n=4 per group); the first group of mice were treated with saline (control), the second group were treated with PP242 (50mg/kg) and the third group were treated with the combination of PP242 50 mg/kg and erlotinib 75 mg/kg. The agents were administrated through oral gavages, twice per week for 21 days. Tumor volumes were measured once every 3 days and calculated based on the formula: V =4/3 x πx (length/2x[width/2]^2^). At the end of treatment, the mice were sacrificed and the tumors were removed and weighed at necropsy.

### Statistical analysis

All data were presented as means ± SE. Statistical analyses were performed by GraphPad Prism version 5.01 software for Windows (GraphPad Software). The differences in the means between two groups were analyzed with two-tailed unpaired Student’s *t*-test. Results were considered to be statistically significant at P <0.05.

RETRACTED

## Results

### PP242 treatment results in a temporal inhibition of AKT phosphorylation

The expression of mTOR, RACTOR, RICTOR, p70S6K and 4E-BP1 is elevated in colorectal carcinoma [44,45]. Because mTORC2 phosphorylates AKT at S473 (AKT^S473^) [9–11], we thought to identify the AKT^S473^ and determine whether the mTORC2 are activated in the carcinoma. Western blotting revealed that AKT^S473^ were elevated in the carcinoma tissues as compared with the matched normal tissues (Figure 1A), thus suggesting the activation of mTORC2 in the carcinomas; however, non-phosphorylated AKT was also elevated, which could not rule out the possibility that the overexpression might cause the phosphorylation in the cancer tissues. During the activation of mTORC1, its substrate p70S6K phosphorylates ribosomal protein S6 [7]. The expression of S6 protein was consistent in matched carcinoma and normal tissues, but detection of the phosphorylated S6 at S235/236 (S6^S235/236^) in the carcinoma but not matched normal tissues suggested the elevated mTORC1 activity in the carcinomas (Figure 1A).

**Figure 1:** PP242 transiently inhibits mTORC2 activity in colorectal carcinoma cells. (A) Western blot analysis for the presence of phosphorylated (p-) and unphosphorylated AKT and S6 in matched colorectal carcinoma tumor (T) and adjacent normal colorectal tissues (N). β-actin was used as protein loading control. The numbers label the cases. (B) The colorectal carcinoma cell lines as indicated were treated with PP242 in the indicated concentrations and then subjected to cell viability assay. The experiment was repeated three times and the data presented as mean + SD (standard deviation). (C) Each of the cell lines as indicated to the top of the panel were untreated or treated with PP242 (1 μM) for the indicated hours and then examined by western blotting using antibodies against the phosphorylated (p-) and unphosphorylated proteins as indicated to the left of the panel.

To determine whether the mTOR kinase inhibitor PP242 block mTORC1 and mTORC2 kinase activity in the carcinoma cells, we first examined a panel of eight carcinoma cell lines for the response to PP242 and showed that PP242 treatment inhibited the growth of each cell line in a dose-dependent manner (Figure 1B). Next, we examined the phosphorylated S6^S235/236^ and 4E-BP1 at T36/45 (4E-BP1^T36/45^) and the mTORC2 substrate AKT^S473^ in the cells after PP242 treatment at the high dose of 1 μM. Western blotting showed that PP242 treatment at the high dose completely abolished the S6^S235/236^ but partially reduced the 4E-BP1^T36/45^ (Figure 1C), consistent with the earlier report that PP242 incompletely inhibits 4E-BP1 phosphorylation [48]. In contrast, PP242 treatment led only to a temporal ablation of the AKT^S473^ in the first few hours of the treatment and the AKT^S473^ gradually returned to the base-line levels as observed in untreated cells within approximately twenty four hours of the treatment (Figure 1C). These data indicate that PP242 can only transiently blocks the mTORC2 kinase activity in colorectal carcinoma cells.

RETRACTED

### PP242 treatment increases EGFR phosphorylation

RTKs activates mTOR kinase through PI3K-AKT pathway [51]; thus to examine whether PP242 treatment may activate RTKs, we treated DLD-1 cells either with rapamycin (0.1 μM) or PP242 (1 μM) for 72 hours and examined the cell lysates for RTK phosphorylation using a RTK phosphorylation array. Interestingly, the array detected phosphorylated EGFR in the cells treated with PP242, but not treated with rapamycin and untreated (Figure 2A). To further examine whether and how rapamycin and PP242 affect the EGFR pathway in the carcinoma cells, the colorectal carcinoma cell lines DLD-1 and HT29 were grown in 1% FBS culture medium containing 50 ng/ml of EGF. Since this experimental design mimics the endogenous EGF-EGFR pathway in the cancer, it is often used in study of the pathway in cancer cells. The cells were treated either with rapamycin or PP242; western blotting showed that the treatment of rapamycin did not affect the levels of either unphosphorylated or phosphorylated EGFR at T1068 (EGFR^T1068^) in the cell lines (Figure 2B); the data indicate that rapamycin did not activate EGFR. Detection of phosphorylated AKT (AKT^S473^) kept in line with the report that rapamycin does not inhibit mTORC2 [22].

**Figure 2:** PP242 treatment leads to the EGFR phosphorylation in the carcinoma cells. (A) RTK arrays of DLD-1 cells untreated or treated with rapamycin (0.1 μM) and PP242 (1 μM) for 72 hours show the phosphorylated EGFR (p-EGFR) as indicated by arrows. (B) DLD-1 and HT29 cells grown in EGF (50 ng/ml) containing medium were treated with rapamycin (0.1 μM), PP242 (1 μM), or LY294002 (20 μM) for the indicated hours and examined by western blotting for the presence of the phosphorylated and unphosphorylated proteins (*left*). (C) DLD-1 and HT29 cells grown in EGF (50 ng/ml) containing medium were treated with PP242 (1 μM) or BKM120 (1 μM) for the indicated hours and tested by western blotting for the presence of the proteins (*left*).

In contrast, the treatment of PP242 led to an increase of the phosphorylated EGFR^T1068^ and AKT^S473^ in a timely manner in both cell lines (Figure 2B). Thus suggests that incomplete inhibition of mTORC2 by PP242 leads to the EGFR phosphorylation and activation. To test whether PP242, like rapamycin, may activate feedback loops through PI3K-mediated AKT phosphorylation [30,31], we treated the cells with the PI3K inhibitor, LY294002 [52]. The treatment of LY294002 failed to inhibit the phosphorylated AKT (AKT^S473^), the substrate of mTOCR2. LY294002 is not selective PI3K inhibitor and, to confirm the role of PI3K, we repeated the experiment with a selective PI3K inhibitor BKM120 [53,54]. The treatment of BKM120, again, failed to inhibit the rebound AKT^S473^ under the PP242 treatment (Figure 2C). Taken together, these results suggest that PP242 treatment increases EGFR phosphorylation through a PI3K independent pathway.

RETRACTED

### The combination of PP242 and erlotinib completely blocks mTORC1 and mTORC2 activity

The parallel increase in EGFR^T1068^ and AKT^S473^ suggests the possibility that the EGFR activation may contribute to the resume of mTORC2 activity in colorectal carcinoma cells under PP242 treatment. To test this notion, we treated DLD-1 cells with PP242 (1 μΜ), alone or in the combination with the EGFR inhibitor, erlotinib (2 μM). The erlotinib treatment blocked the phosphorylation of EGFR, temporally inhibited S6 phosphorylation but had no effect on 4E-BP1 phosphorylation (Figure 3A). In contrast, the combination treatment blocked the phosphorylation of EGFR (EGFR^T1068^) and mTORC1 substrates (S6^S235/236^; 4E-BP1^T36/45^); thus, EGFR activation contributes to the incomplete inhibition of mTORC1 by PP242 and in combination with the EGFR inhibitor erlotinib, PP242 can completely block the mTORC1 kinase activity. The treatment of PP242 (Figure 2B) and erlotinib (Figure 3A) alone did not affect the p-AKT; but the combination treatment ablated the p-AKT (Figure 3A). The data suggest that the inhibition of p-AKT is due to the synergistic effects; however, the mechanism remains to be elucidated.

**Figure 3:** The combination of P242 and erlotinib inhibits the carcinoma cell growth. (A) DLD-1 cells grown in EGF (50 ng/ml) containing medium were treated with erlotinib (2 μM) and PP242 (1 μM), alone or in combination, for the indicated hours and analyzed by western blotting for the indicated proteins (*left*). (B) DLD-1 and HT29 cells were treated with PP242 (1 μM) and erlotinib (2 μM), alone or in combination, and then subjected to cell viability assay. The data were presented as mean + SD. **, p < 0.01. (C) Colony formation assay of DLD-1 cells, treated or untreated with PP242 (1 μM) and/or erlotinib (2 μM), shows the colony densities in culture wells. (D) The colony numbers from the colony formation assay as described above in C were accounted and presented as mean + SD. NS, no significance; **, p < 0.01.

RETRACTED

Next, we thought to examine the biological effects of the combination of EGFR and mTOR inhibitors on colorectal carcinoma cells. To this end, we treated the carcinoma cell lines with erlotinib (2 μM) and PP242 (0.5 μM), alone and in combination, for 24 hours in the presence of EGF (50 ng/ml) according to the experimental design as described in Figure 2. Cell viability assay revealed that the combination treatment produced a significant synergy in the cell growth inhibition (Figure 3B). To examine this further, we treated the cells for 14 days in a colony formation assay and showed that the combination treatment synergistically eliminated the formation of colonies from each of these cell lines (Figure 3B, C). Collectively, these results suggest that the combination of PP242 and erlotinib completely blocks both mTORC1 and mTORC2 kinase activity and synergistically inhibits the growth of colorectal carcinoma cells.

### The combination of PP242 and erlotinib induces apoptotic cell death

PP242 has been reported to induce apoptosis in leukemia and breast cancer cells through inhibition of mTORC2 activity [42,43]. The combination of P242 and erlotinib can inhibit the mTORC2 activity, which suggests that the combination may induce apoptosis in colorectal carcinoma cells. To text this notion, we treated DLD-1 cells with PP242 (0.5 μM) or erlotinib (2 μM), alone and in combination in the presence of EGF (50 ng/ml). Flow cytometry detected approximately 5% sub-G1 apoptotic cells in the cells treated with PP242 or erlotinib alone (Figure 4A). In contrast, approximately 15-20% cells underwent apoptotic cell death under the combination treatment of PP242 and erlotinib (Figure 4A). To confirm the PP242 and erlotinib combination-induced apoptosis, we examined the treated cells on western blotting and thus revealed cleavage of caspase-3, DFF45 and PARP; the data confirmed the apoptotic cell death of the cells under the treatment of PP242 and erlotinib, in contrast, however, PP242 and erlotinib alone failed to induce apoptosis in the cells (Figure 4B). These results suggest that the combination of PP242 and erlotinib synergistically inhibits the growth of colorectal carcinoma cells in part through induction of apoptosis.

**Figure 4:** PP242 and erlotinib treatment induce apoptotic cell death. (A) DLD-1 cells were treated with erlotinib (2 μM) and PP242 (1 μM), alone or in combination, for the indicated hours and then analyzed by flow cytometry. The percentage of sub-G1 apoptotic cells were presented as mean + SD. **, p < 0.01. (B) DLD-1 cells were treated with PP242 (1 μM) and/or erlotinib (2 μM) for the indicated hours and analyzed by western blotting for the cleavage of caspase-3, DFF45 and PARP with the molecular weights of the cleavage products indicated to the right of the panel.

RETRACTED

### Combined PP242 and erlotinib treatment suppresses colorectal carcinoma xenografts

To evaluate therapeutic potential of the combination of PP242 and erlotinib in treating colorectal carcinoma, we generated subcutaneous xenografts by injecting subcutaneously DLD-1 cells in athymic (nu/nu) mice. Once the xenografts were formed at approximately 150-200 mm^3^ sizes, the mice were treated for 21 days through oral gavage of saline as control or PP242 (50mg/kg), alone or in combination with erlotinib (75 mg/kg). Our earlier work [55] and the data presented in Figure 2 have shown that erlotinib treatment alone has no effects on DLD-1 cell growth and, thus, we omitted erlotinib treatment alone and saved a group of mice. Tumor volumes were measured once every 3 days and mice were followed closely for 21 days. The results showed that the combination of PP242 and erlotinib significantly enhanced the therapeutic effects of PP242 treatment (Figure 5A). At necropsy, the significant difference in the tumor sizes was observed among the three groups of mice (Figure 5B). The tumors were removed and the tumor weights further indicated the significant synergy of the combination treatment (Figure 5C). Western blotting of fresh tumor tissues showed that the combination treatment abolished the mTORC1 substrate, S6^S235/236^ and the mTORC2 substrate AKT^S473^. Collectively, these results indicate that the combination treatment of PP242 and erlotinib completely blocks the mTORC1 and mTORC2 kinase activity, induce apoptosis in colorectal carcinoma cells and suppresses the carcinoma xenograft progression.

**Figure 5:** PP242 and erlotinib treatment suppresses xenograft progression in mice. (A) DLD-1 cells were injected subcutaneously in mice for xenograft formation and then treated with oral gavage of saline in control group of mice, PP242 in monotherapy, and PP242 plus erlotinib in combination treatment for the indicated days. The tumor volumes from the same group mice were grouped and presented as mean + SD. (B) At necropsy, the representative mice bearing subcutaneous xenografts were shown from the left to the right with PP242 and erlotinib combination, PP242 alone and saline. (C) The xenografts were dissected from mice and their weights were presented mean + SD. *, p < 0.05; **, p < 0.01. (D) The xenografts were lysed and subjected to western blotting for the presence of phosphorylated and unphosphorylated proteins in the xenograft tissues.

RETRACTED

## Discussion

Emerging evidence supports the notion that targeting of mTOR pathway may provide effective treatment of colorectal carcinoma [2]. Immunohistochemistry shows the elevation of the mTOR pathway proteins such as mTOR, RACTOR, RICTOR, p70S6K, eIF4E and 4E-BP1 in human colorectal carcinoma tissues [44–46]. Knockdown of mTOR protein by RNA inferring inhibits the carcinoma growth [45]. However, phase I and II clinical trials of the first generation of mTOR inhibitors have shown limited if any clinical benefit in treating colorectal carcinomas as signal agents [2,56]. Mechanistically, the cancer resistance to the treatment is mainly because rapalogs incompletely inhibits mTORC1 and do not inhibit mTORC2 and thus activate both PI3K/AKT and ERK cell growth pathways through negative feedback loops [56].

In contrast, the second generation of mTOR inhibitors targets the mTOR kinase activity, thus inhibits both mTORC1 and mTORC2 and are more potent than the first generation of the inhibitors [22]. While the ongoing clinical trials will determine whether these mTOR kinase inhibitors are effective in clinical treatment of colorectal carcinomas, preclinical study of the carcinoma cell lines reveals the resistance of many of the cell lines to the treatment of the mTOR kinase inhibitor PP242 in part due to mTOR-independent 4E-BP1 phosphorylation [48]. Consistent with this earlier finding, we show here that PP242 treatment leads to the incomplete inhibition of 4E-BP1 phosphorylation in colorectal cells. 4E-BP1 is a key effector of the PI3K and mTOR pathway [57] and the incomplete inhibition by PP242 of the 4E-BP1 phosphorylation contributes to the carcinoma resistance to PP242 treatment [48].

The results reported here indicate that PP242 only transiently inhibits mTORC2 kinase activity in colorectal carcinoma cells. Early studies show that PP242 treatment inhibits the AKT phosphorylation at S473 (AKT^S473^), the mTORC2 phosphorylation site on AKT, in colorectal carcinoma cells at 12 hour [48] and pancreatic carcinoma cells at 2 hour of the treatment [34]. In a time course experiment, however, we show that the phosphorylation of AKT^S473^ resumes gradually up to the untreated cell levels within 24 hours of PP242 treatment and inhibition of PI3K fails to block the AKT^S473^ phosphorylation. In contrast, rapamycin does not inhibit the AKT^S473^ phosphorylation through the time course, keeping in line with the notion that rapamycin does not inhibit mTORC2 activity [34]. Our results demonstrate for the first time that the second generation of mTOR kinase inhibitor PP242 can inhibit mTORC2 activity but the inhibition is incomplete and transient in colorectal carcinoma cells.

RETRACTED

Another salience of our results is that PP242 treatment leads to the increase of EGFR phosphorylation through PI3K-independent pathway in colorectal carcinoma cells. EGFR can activate downstream PI3K and ERK pathway and thus drives cancer progression [58]. While it remains to be investigated, recent findings that PP242 treatment activates ERK pathway in multiple myeloma [59] and pancreatic carcinoma cells [34] suggest the possibility that the mTOR kinase inhibitor PP242 may activate ERK pathway through the EGFR activation. The feedback activation of PI3K-AKT and ERK pathway undermine the usefulness of the first generation of mTOR inhibitors in clinical treatment of cancers. The data presented here in study of colorectal carcinoma, together with the data in studies of myeloma and pancreatic carcinoma cells suggest the presence of feedback activation of ERK for the second generation of mTOR kinase inhibitors perhaps due the incomplete inhibition of mTORC2 activity and thus raise the concern on whether PP242 is effective in clinical treatment of cancers as single agents.

The study presented here provides several lines of evidence in support of the notion that the combination of mTOR kinase and EGFR inhibitors may provide strategy in treatment of colorectal carcinoma. First, the combination treatment of erlotinib and PP242 results in the complete inhibition of mTORC1 and mTORC2 activity in the carcinoma cells. Second, the combination inhibits the colony formation and cell growth. Thirdly, the EGFR inhibitor enhances PP242-induced apoptosis. Finally, erlotinib enhances PP242 therapeutic efficacy in treatment of colorectal carcinoma xenografts. EGFR has been therapeutic targeted by small molecular inhibitors and neutralizing antibodies [60]; however, these EGFR inhibitors have failed to show clinical benefits in treating colorectal carcinoma [61,62]. The mechanisms of cancer resistance to EGFR inhibitors include the activation of redundant downstream kinase pathways; thus, there is a need for combination therapies targeting these redundant pathways [63].

Phase I and II trials of erlotinib have created controversial regarding the toxicity of the agent. As a single agent, erlotinib was tolerated by patients in phase I trial of treatment of metastatic colorectal carcinoma [64]. Phase II trials of erlotinib, either in combination with multiple agents (5-fluorouracit, leucovorin, oxaliplatin, bevacizumab) or with capecitabine have shown the toxicity of these combination regimens in treating patients with metastatic colorectal cancer [65,66]. In the meantime, however, three clinical trials have failed to show the toxicity of erlotinib in combination with capecitabine and oxaliplatin [67], capecitabine and irinotecan [68], and cetuximab in the treatment of metastatic colorectal carcinoma [69]. While only clinical trials will determine whether the combined erlotinib and PP242 treatment can be tolerated by patients, our preclinical study here provides the rational for clinical trials of the combination of mTOR kinase and EGFR inhibitors for treatment of metastatic colorectal carcinoma.
